This article has been retracted.

# The Use of Internet of Things and Cloud Computing Technology in the Performance Appraisal Management of Innovation Capability of University Scientific Research Team

**DOI:** 10.1155/2022/9423718

**Published:** 2022-04-10

**Authors:** Siyu Meng, Xue Zhang

**Affiliations:** College of Business Administration, Liaoning Technical University, Huludao, Liaoning 125105, China

## Abstract

This study aims to speed up the progress of scientific research projects in colleges and universities, continuously improve the innovation ability of scientific research teams in colleges and universities, and optimize the current management methods of performance appraisal of college innovation ability. Firstly, the needs of the innovation performance evaluation system are analyzed, and the corresponding innovation performance evaluation index system of scientific research team is constructed. Secondly, the Internet of Things (IoT) combines the Field Programmable Gate Array (FPGA) to build an innovation capability performance appraisal management terminal. Thirdly, the lightweight deep network has been built into the innovation ability performance assessment management network of university scientific research teams, which relates to the innovation performance assessment index system of scientific research teams. Finally, the system performance is tested. The results show that the proposed method has different degrees of compression for MobileNet, which can significantly reduce the network computation and retain the original recognition ability. Models whose Floating-Point Operations (FLOPs) are reduced by 70% to 90% have 3.6 to 14.3 times fewer parameters. Under different pruning rates, the proposed model has higher model compression rate and recognition accuracy than other models. The results also show that the output of the results is closely related to the interests of the research team. The academic influence score of Team 1 is 0.17, which is the highest among the six groups in this experimental study, indicating that Team 1 has the most significant academic influence. These results provide certain data support and method reference for evaluating the innovation ability of scientific research teams in colleges and universities and contribute to the comprehensive development of efficient scientific research teams.

## 1. Introduction

Research teams are generally closely related to national laboratories or school laboratories. Team leaders are mainly responsible for the guidance of high-level fundamental research and applied fundamental research. Research teams in universities are composed of laboratories, generally composed of teachers and students, based on teaching departments and research departments that are responsible for related scientific research projects. In the existing Chinese system, universities are responsible for fundamental research, innovative research, and talent introduction and training. National science and technology construction is related to the competitiveness of universities. However, there are some problems in colleges and universities in China, such as poor concentration of related resources, low financial resources, and difficult interdisciplinary cooperation. At present, the construction of research teams in universities is gradually strengthened with considerable investment of material and financial resources [1]. Under the current situation, it has become an unavoidable problem to conduct exploratory research on the university scientific research team innovation to help the reasonable operation, benign development, and competitiveness improvement of universities. With the accelerating pace of global economic integration, scientific and efficient performance management system and assessment system become more important in promoting the development of scientific and technological innovation in universities. IoT has made good progress in many fields and realized intelligent management in related fields. IoT is considered to be a revolutionary and innovative technology to accelerate industry informatization and realize the transformation of traditional industries. Broadly speaking, IoT is the integration and interworking of information space and physical space. Digitization, networking, automation, and intelligence of everything around people are not only an effective means to realize efficient information exchange but also a higher level of comprehensive application of informatization in human society. With the development of industrialization and the attention of universities and education departments to the performance appraisal management of innovation capability of university scientific research teams, IoT is gradually being introduced into the field of performance appraisal management. Moreover, intelligent edge computing is widely used in IoT applications, especially in scenarios with special business requirements such as low delay, high bandwidth, high reliability, massive connection, heterogeneous aggregation, and local security and privacy protection. The combination of IoT and Digital Twins (DTs) is also excessively practical. DTs makes full use of physical models, sensor updating, operation history, and other data and integrates multidisciplinary, multiphysical quantity, multiscale, and multiprobability simulation process to map and reflect the whole life cycle process of physical equipment in virtual space. In the intellectualization process via IoT, intelligent edge computing combined with DTs technology is a quite reliable path, which can realize multiple intellectualization cases, such as intelligent manufacturing, intelligent city, intelligent transportation, and intelligent furniture. Similarly, the integration of intelligent edge computing and DTs technology can effectively support the performance appraisal management of innovation capability of university scientific research teams.

To sum up, the combination of intelligent edge computing and DTs technology evaluates the innovation ability of university scientific research teams, aiming to provide more scientific and predictable evaluation and management information for management decisions of university managers. There are two aspects of innovation: (1) The scientific research team is regarded as a whole. Quantitative evaluation methods are used to evaluate the innovation performance of existing university scientific research teams. The corresponding evaluation theory is perfected. (2) In view of the limitation of computing resources in the edge environment, two compression algorithms are used to reduce the model parameters and the amount of computation based on transfer learning and training the MobileNet model. Results are analyzed based on data obtained from questionnaires and open databases. Furthermore, simulation learning is used to recover the recognition accuracy. A deeply compressed edge end model is obtained.

## 2. Literature Review

At present, scholars have carried out research on teaching performance evaluation in colleges and universities. Chen evaluated the teachers' teaching performance level in some educational courses from the perspective of ordinary education diploma students. They adopted the descriptive analysis method and designed a questionnaire to evaluate teachers' teaching performance. The research results showed that, from the perspective of general education diploma students, the teaching performance of teaching staff was relatively high. Students' evaluation of teachers' performance was general after teaching. Besides, there was no significant difference in students' evaluation among different ages and professional curriculum. There only existed differences in evaluation methods and feedback of senior students [2]. Praus pointed out that it was significant for provincial key laboratories to summarize experiences, discover problems, bridge the gap and weakness, and improve sci-tech strength through assessment and evaluation. However, the current evaluation indicator system still had an obvious “four-only” tendency, which was difficult to objectively evaluate the development of key laboratories. Based on the principle of whole process management, the author constructed an evaluation indicator system for disciplinary, enterprise established and provincial-municipal coconstructed provincial key laboratories from three dimensions of “quantity,” “quality,” and “effectiveness” and used the best-worst method to determine the weight of indicators at all levels. The “quantity,” “quality,” and “efficiency” indicator system can scientifically reflect the performance of provincial key laboratories, improve the shortcomings of the previous “four-only” evaluation, and provide reference for its subsequent development and optimization [3]. Kim and So conducted the evaluation on the performance of a small group of 49 young scholars, such as doctoral students and postdoctoral and junior researchers, working in different technical and scientific fields, based on 11 types of research outputs. Principal Component Analysis was used to statistically analyze the research outputs and its results were compared with factor and cluster analysis [4]. Xia et al. established a scientific evaluation index system of student portraits to effectively evaluate the academic performance of university students under the context of significant changes in all aspects of education under big data. They took an object-oriented programming course as an example and collected various data of university students' academic performance. The collected data was normalized and the weight of each evaluation index was determined by Analytic Hierarchy Process (AHP). Then, the authors constructed a fuzzy evaluation model based on big data to evaluate the various dimensions of university students' academic performance. Evaluation results revealed the problems of university students in learning and practice, helped to shape the image of each student, and promoted the realization of personalized education [5].

In recent years, Convolutional Neural Networks (CNN) have achieved great success in the field of computer vision, such as image classification and object detection. However, due to the limitation of storage space and computation, the application of CNN in embedded and mobile devices with certain storage and computation requirements is still a big challenge. Therefore, compressing models to reduce storage space and computational consumption has become a research hotspot. Kim et al. [6] proposed that automatic modulation classification in cognitive radio networks is a key method for efficient use of spectrum resources. However, traditional likelihood-based methods have high computational complexity. Therefore, they proposed a novel Convolutional Neural Network structure that adopts an asymmetric convolutional structure to reduce the computational complexity. Furthermore, they solved gradient vanishing to improve classification accuracy using skip connection technique. Wang et al. [7] pointed out that automatic modulation classification is a noncooperative communication system technology suitable for military and civilian scenarios. They proposed a lightweight automatic modulation classification method based on deep learning. The model size of this method is smaller and the calculation speed is faster. In this method, the authors introduce a scaling factor for each neuron in the neural network and enhance the sparsity of this scaling factor through compressed sensing. Their experimental results show that this method can effectively reduce the model size, speed up the calculation, and reduce the performance loss. Chiu et al. [8] pointed out that the development of real estate price prediction systems is one of the top concerns for researchers. However, most of the existing studies only consider temporal or spatial features and cannot consider both simultaneously, resulting in the problem of prediction accuracy. Therefore, the authors propose three ideas to overcome these problems. (1) They designed a new spatiotemporal data structure, called spatiotemporal influence graph, to quantify the impact of changes in surrounding facilities on housing prices. (2) They designed a new Convolutional Neural Network-Long Short-Term Memory (CNN-LSTM) model for real estate price prediction. (3) They designed a new framework to extract the most important features of a specific type of real estate prices. These features are combined with a shallow recurrent neural network for modeling. The computational complexity of this model is much lower than that of the CNN-LSTM model, which is suitable for practical applications.

Based on the above analysis, Europe, America, and other developed countries have played a pioneering role in the establishment and improvement of performance theory, which has been applied to various fields of university scientific research management from different perspectives. Nevertheless, due to different national conditions, performance evaluation index systems of scientific research management in colleges and universities proposed by European and American researchers cannot be directly applied to scientific research management in colleges and universities in China. Therefore, Chinese domestic scholars usually put forward corresponding performance index systems considering the current situation and problems of the college system in China. However, quantitative thinking and quantitative model are rarely used to analyze the performance of scientific research teams in colleges and universities. In view of the shortcomings existing in previous work, the present work adopts the following methods: The first is literature research method: reference materials for writing are collected from libraries, journals, networks, and statistical yearbook databases, including statistical data, charts, and documents; other research methods and achievements of other scholars are also referenced. The second is statistical analysis method: it refers to a research method to understand and reveal the relationship between things, the law of change, and the development trend of things through the analysis and study of the quantitative relationship of the size, speed, scope, and degree of the research object. It aims to achieve the correct explanation and prediction of things. The third is AHP: it is a decision-making method that disintegrates the elements always related to decision-making into the levels of objectives, criteria, and schemes and conducts qualitative and quantitative analysis on this basis to study the performance appraisal management of innovation capability of university research teams.

## 3. Innovation Performance and Construction of Appraisal Index System

### 3.1. Overview of Innovation Performance of University Research Teams

Innovation performance refers to the comprehensive evaluation of innovation programs, activities, innovation management, and innovation performance management in a specific context, which belongs to economic concepts. Related researchers believe that, on the one hand, innovation performance management can be regarded as an assessment and summary of previous management. On the other hand, innovation performance management can be regarded as the premise of finding and solving problems [9]. When the functions of universities become increasingly complex, scientific research activities in universities have been difficult to be summarized by the research category of science and technology. They have already belonged to the application category of scientific research achievements and technical services. Scientific research performance appraisal is the official measurement and evaluation of scientific and technological innovation activities of researchers, which reveals the effectiveness of researchers' work and the potential evaluation of future work [10, 11]. Research team in local universities is a new type of scientific research institution in local universities with specific particularity. The performance appraisal method of research teams in universities is different from that of other organizations. There are significant differences between university research teams and ordinary social organizations or institutions: The first is clear research objectives. All members of a university research team have clear and united research objectives reflecting the direction of their scientific research [12, 13]. The second is effective academic leaders. Academic leaders in research teams will have a certain impact on the research activities and psychology of team members with their excellent research attitudes and professional accomplishments, thus forming a better research atmosphere. The third is complementary members. Each member of the team is complementary to the others. They have relatively close research level and scientific background, while they play their own expertise in different professional fields. With this framework, university research teams can play their advantages. The fourth is the incentive and constraint mechanism within the team. There are great differences in the constraint and incentive mechanism between university research teams and other institutions. Generally, members of research teams have high comprehensive quality and a strong sense of honor and responsibility, and they generally pursue life value, personal honor, and scientific research achievements. Therefore, the incentive and constraint mechanism has an obvious incentive effect [14, 15].

Due to the diversification of the development of science and technology, there is a certain degree of integration between various disciplines, so it is difficult to distinguish the specific category of research. Under the current situation of China, each university has different development, and its scientific research achievements also match its development stage. Generally, the innovation performance of research teams in universities is evaluated from the three following points: The first is academic influence level. The scientific research status and research strength of different universities are distributed according to the meetings participated in by research teams and their positions. The second is the quality and number of scientific research achievements. A team's scientific research achievements emphasize whether a team publishes articles in critical journals. The third is framework composition of scientific research personnel. Objective factors are the key points such as educational background and title of scientific research personnel within a team [16–18].

Among the emerging performance appraisal methods, the most common are peer review, AHP, balanced scorecard, and fuzzy comprehensive evaluation. Peer review refers to assessing academic achievements by experts and scholars in the same field. Still, only educational theories and practical tests are the absolute measurements of academic standards. The meanings of peer review and academic standards are different. The balanced scorecard method originated from the “measurement of future organizational performance evaluation system” proposed by a professor at Harvard University. It implements organizational strategies from four perspectives: operational indicators, target value finance, customers, and internal functional learning and growth. However, the balanced scorecard method also has its defects. It is only applicable to the performance management scenario that focuses on financial indicators. A fuzzy comprehensive evaluation can achieve the goal of combining quantitative and qualitative factors, which is commonly used to evaluate the complete state of transactions [19, 20].

### 3.2. Construction of Innovation Performance Appraisal Index System for Research Teams

With the continuous progress of science and technology in China, research teams in universities have gradually become the backbone of innovative science and technology. Therefore, universities should pay attention to the construction of research teams, improve the professional and technical level of research teams, and give full play to the scientific research potential of teams. Performance appraisal is an important measure specially used to evaluate team efficiency, which can help relevant researchers clearly understand research teams' actual scientific research strength [21, 22]. Therefore, research management departments in universities need to pay attention to the performance appraisal management of research teams. Correspondingly, an innovation performance index of university research teams is constructed, through which the research status of each member is analyzed of a research team. It is found that there are some problems in the innovation performance appraisal of university research teams. (1) The innovation appraisal system is not perfect. The current innovation performance appraisal method of research teams often focuses on the evaluation and management of the team. When conducting performance appraisal, it generally only evaluates the research results of scientific research projects, the number of awards, and the situation adopted by the government. Universities often only value the work and contribution of the leading project leaders but ignore the contribution and work of other team members, resulting in a certain degree of damage to these members. They may consider their work as unrecognized, which reduces their research enthusiasm. (2) The appraisal mechanism is unscientific. At present, most university research teams still adopt the overall appraisal method focusing on task completion. There are certain differences in the value of each member's work content and contribution to a team. There is no appraisal of the group members' necessity in the scientific research tasks, making it difficult for team managers to provide necessary performance rewards [23, 24].

Based on the above analysis, there is a lack of a comprehensive and universal appraisal index system with guiding significance in universities. The index system used in most schools now mainly has two problems. Firstly, there are intersections between the same level of indexes. Secondly, the selection of indexes does not match the actual situation of university research teams. Therefore, the innovation performance index system is optimized for university research teams. Finally, the preliminary appraisal index system is designed, as shown in Figure 1.

Since the number of researchers in local universities is large, the corresponding data is normalized as shown in the following equation:

(1) $$\begin{array}{c} y\left(k\right)=\;\log_{10}\left(x\left(k\right)\right),\;k=1,2,\ldots ,N. \end{array}$$

In equation (1), *x* represents the number of talents selected by universities, and *N* denotes a positive integer.

Quantitative indexes cannot directly realize the appraisal of scientific research innovation in universities. Additionally, the AHP can combine quantitative and qualitative analysis and produce conclusions based on influencing factors [25, 26]. Therefore, the AHP is adopted to study the weight coefficient with four steps. The first step is to build a hierarchical ladder model. The second step is to solve the judgment matrix. The third step is to calculate the single-level index weight, and the fourth step is to calculate the weight value of the total-level index.

During the construction of the hierarchical ladder model, the target layer of the innovation performance appraisal system is set as *A*, with the criterion layer as *B*, the academic influence in the criterion layer as *B*_1_, the successful output as *B*_2_, the talent cultivation as *B*_3_, the subcriterion layer as *C*, and the bottom layer of the index layer as *D*. The working principle of AHP is to use the primary data of information to judge each layer element in the matrix and analyze the importance of the data. After comparison, the final judgment matrix is formed, and then the consistency of the matrix is judged to obtain the vector closest to the weight [27].

Based on the above, it can be found that different influencing factors have other impacts on the overall effect of innovation performance, and the performance appraisal index has a particular effect on the weight of the final index. Thus, APH is used to determine the index weight value to obtain better appraisal results of the performance index, with the determination of the index weight at the same level by the knowledge and experience of experts. The importance of some indexes obtained in the experiment is shown in Figure 2.

### 3.3. Intelligent Edge Computing

With the continuous development of IoT technology and big data technology, the connection between IoT technology and big data technology has become increasingly close. The amount of data to be processed by equipment has proliferated, promoting the generation and development of edge computing models. The core of edge computing technology is to change the execution center of computing tasks. In other words, some computing tasks on cloud service centers are unloaded to the edge equipment with enhanced computing ability to complete so that the processing load of the cloud service center is reduced, the congestion of the network is alleviated, and the task processing efficiency is improved [28, 29]. As a new calculation model, the processing objects of edge calculation are divided into the data generated by the downlink tasks in cloud services and the data generated by the uplink tasks in IoT services. Edge computing is a distributed computing model with storage, calculation, and network capabilities in the actual scene. This computing model mainly deals with the data generated by edge devices in work and makes the devices with data processing capabilities close to the edge of the user's mobile network to provide users with better and more efficient edge intelligent services [30, 31] to improve service quality and user satisfaction. The IoT, mobile extensive data analysis, and the Internet of Vehicles are common application scenarios of mobile edge computing [32, 33]. Compared with the traditional cloud computing technology, edge computing has four advantages: (1) short response delay, (2) high security and privacy, (3) low communication overhead, and (4) robust scalability. Based on the above analysis, edge computing can respond quickly to the user's business needs on the data side and reduce the dependence of the service on the wireless network so that it can still provide essential services for users without a network. Besides, edge computing processes data locally, which greatly guarantees the security and privacy of user information [34–36]. Based on the above analysis, edge computing, as the evolution and development of cloud computing technology, has the characteristics of close application, intelligence and flexibility, and efficient distribution. It has a broad application prospect in IoT, industrial manufacturing, and transportation. Mobile edge computing mainly solves the problem of traditional mobile cloud networks. Mobile edge computing uses the edge of the user's mobile terminal to complete the calculation task and uses distributed methods to perform edge big data processing [37, 38].  Figure 3 reveals the three parts of the edge computing system, which carry out edge computing in different ways to improve efficiency.

In Figure 3, with the rapid development of mobile devices, various mobile platforms are also trying to complete multiple complex logical functions, such as large-scale games and smart tools that are more dependent on resources. However, low-performance batteries limit the application scenarios and programs of mobile devices and affect user experience. Mobile edge computing provides a solution to the energy consumption of mobile devices. Therefore, mobile edge computing systems continue to emerge. It mainly refers to the establishment of a remote computing service system consisting of a large number of servers outside the user equipment. Then, the user offloads the task data that needs to be calculated to the mobile edge computing system and provides the user with a remote and efficient computing service through its efficient computing service, thereby reducing the utilization rate of the user equipment. It integrates different resources in the cloud and expands the hardware performance of mobile devices by linking the cloud and mobile terminals. When computing offload is required, the mobile device uses cloud resources to transfer the workload of the mobile application to the cloud for collection, thereby reducing the energy consumption of the mobile device. Therefore, intelligent edge computing can work in various situations, saving resources. In addition, it has a wide range of applications and multiple advantages. This work innovatively uses intelligent edge computing to evaluate the innovation ability performance of colleges and universities, which can effectively improve the efficiency of the innovation ability performance evaluation management of scientific research teams in colleges and universities.

## 4. Network Design of Performance Appraisal of University Scientific Research Team

Deep neural networks have been proven effective in solving problems in different fields such as image and natural language. Meanwhile, with the continuous development of mobile Internet technology, portable devices have been popularized rapidly, and users put forward growing needs. Therefore, designing an efficient and high-performance lightweight neural network is the key to solving the problem. At present, the main idea of the artificial design of lightweight neural networks is to design more efficient network computing methods. The lightweight CNN MobileNet is selected as the benchmark model of this study. MobileNet model decomposes the traditional convolution into a deep convolution and a 1 *∗* 1 point-to-point convolution with a convolution kernel. The calculation speed is 8∼9 times faster than the conventional convolution. It is mainly for high-end embedded systems such as smartphones. To deeply compress MobileNet, an edge computing-oriented performance evaluation management method is proposed for the innovation ability of university scientific research teams, as shown in Figure 4.

In the first stage of the method, the MobileNet model trained by channel pruning compression migration learning is used. Compared with training from scratch, transfer learning can effectively improve the recognition accuracy of the model. Transfer learning initializes the model with the pretrained parameters on the ImageNet dataset. It then optimizes the model parameters through the standard multiclassification loss function on the dataset collected here. Finally, channel pruning based on the *L*_1_ norm reduces the lightweight convolution kernel. The pruned model is further compressed by a quantitative method to obtain a lightweight edge model in the second stage. Through quantization, the weight and activation of the model are reduced from 32 bits to 8 bits, divided into quantization during training and quantization after training. Although the quantization during training is more suitable for lightweight models, directly using this method to compress the pruned MobileNet model will still lead to a significant decline in recognition accuracy. Therefore, simulation learning is combined with quantization during training in the second stage. The MobileNet of transfer learning is used to supervise the quantization training process of the pruned model to realize quantitative simulation learning and improve the recognition accuracy while compressing the model.

Model channel pruning uses the uniform pruning method to prune the separated convolution layer of the MobileNet model; in other words, each layer subtracts the convolution kernel of the same proportion. The pruning ratio of each layer is determined according to the need to reduce the number of Floating-Point Operations (FLOPs) of the model. The convolution kernels in each layer are sorted from high to low *L*_1_ norm, and the convolution kernels with inferior *L*_1_ norm are pruned first, and the convolution kernels with low *L*_1_ norm are pruned first. To realize the deep compression of the model, a higher proportion of channel pruning is required, and 70%, 80%, and 90% of FLOPs are reduced for the model, respectively. Quantitative simulation learning uses the simulation learning loss function as the quantitative loss function during training. The simulation learning method makes the output characteristics of the model after pruning and quantization as close as possible to the MobileNet output characteristics of transfer learning training. The *L*_2_ norm between the two output characteristics is used as the analog loss function, as shown in the following equation:

(2) $$\begin{array}{c} L_{L_{2}}\left(W_{s},W_{t}\right)={\left\|F\left(x;W_{t}\right)-F\left(x;W_{s}\right)\right\|}_{2}^{2}. \end{array}$$

In equation (2), *W*_*t*_ and *W*_*s*_ mean the weight matrix of MobileNet trained by transfer learning and the model after pruning quantization, *F*(*x*; *W*_*t*_) represents the output eigenvalue of the MobileNet model, and *F*(*x*; *W*_*s*_) denotes the output eigenvalue of the model after branch quantization.

After pruning and quantization, the output characteristics of the model are normalized by Softmax to obtain the prediction category probability. After comparison with the classification label, cross-entropy is accepted as the standard multiclassification loss function *L*_class_(*W*_*s*_). The complete loss function of simulation learning is the weight of classification loss function and simulation loss function, as presented in the following equation:

(3) $$\begin{array}{c} L\left(W\right)=L_{\text{class}}\left(W_{s}\right)+\alpha L_{L_{2}}\left(W_{s},W_{t}\right). \end{array}$$

In equation (3), *α* refers to the hyperparameter of balancing loss weight.

The quantization during training is combined with simulation learning to realize quantitative simulation learning. The specific training steps are as follows:

Step 1: In the forward propagation of training, the weight *w*_*f*_ and activation *a*_*f*_ of the model are quantized to obtain the fixed-point value *w*_*q*_ and *a*_*q*_. For the floating-point number *x*, the specific quantization process is shown in the following equation:
  (4) $$\begin{array}{c} x_{\text{int}}=\mathrm{round}\left(\frac{x}{\Delta }\right),\\ x_{Q}=\mathrm{clamp}\left[-\left(\frac{N}{2}-1\right),\frac{N}{2}-1,\;x_{\text{int}}\right]. \end{array}$$
In equation (4), *x*_*Q*_ denotes the obtained quantized value.
Step 2: Calculate the loss function of simulated learning of MobileNet trained by transfer learning after pruning and quantization.
Step 3: In the backward propagation process, the loss function value obtained in Step 2 is used to calculate the gradient of the quantized weight, which can be written as in the following equation:
  (5) $$\begin{array}{c} \frac{\partial L\left(w_{q}\right)}{\partial w_{q}}. \end{array}$$
Step 4: The gradient calculated in Step 3 is used to update the floating-point value before quantization, that is, to inverse-quantize the weight of the model back to the floating-point type with error, as shown in the following equation:
  (6) $$\begin{array}{c} w_{\text{f}}=w_{\text{f}}-v\frac{\partial L\left(w_{q}\right)}{\partial w_{q}}, \end{array}$$
*v* is the learning rate and *f* is a floating point.
Therefore, the backward propagation process of the model is still floating-point calculation.
Step 5: Repeat Steps 1 to 4 until the training is completed. Finally, the model is quantified according to Step 1 to obtain the final edge model.

### 4.1. Construction of Performance Evaluation Management System of Innovation Capability Based on Internet of Things

The IoT-based performance evaluation management system of innovation capability includes a performance management evaluation terminal based on Field Programmable Gate Array (FPGA), which collects and monitors innovation capability performance evaluation information. The module is connected with the antenna through an RF cable and associated with the face recognizer through the Controller Area Network (CAN) bus. The cloud server based on the new assessment principle includes cloud service, user login module, external environment analysis module, internal environment analysis module, and performance index module used to provide performance index decomposition information for the school management according to the internal data of the school and the data collected by the performance management assessment terminal based on FPGA. The system also includes the indicator calculation terminal system of performance appraisal, which is used to determine the weight of indicators. Relevant managers use the remote management control terminal to manage the system. The system's performance management evaluation terminal based on FPGA is connected with the performance mobile terminal through a 5G wireless network mode. It interacts with the cloud server through a 5G wireless network, and the cloud server in the system is connected with the remote management terminal through the network cable.

### 4.2. Design of Data Acquisition Module Based on the Edge Device

According to the design objectives, the system should be suitable for biological data collection scenarios and network data collection scenarios. Therefore, in the design of the data collection module, the functions in the corresponding situations are designed, respectively. Based on the setting of the system structure and the consideration of the actual work scene, the physical data collection module uses the communication scheme between edge equipment and external equipment as the data transmission mode to control the data acquisition state of various sensors. On this basis, the physical data collection is completed. On the one hand, edge devices in the data collection module need to provide cloud computing interfaces and data preprocessing interfaces. The module of coordination with other functional modules and the sensor collected data. On the other hand, it also sends the sensor's existing state and control function to the cloud to grasp the cloud computing center for the actual collection status. In the network data collection scene, the system uses multiple edge devices to work together under the unified command of the cloud center. Besides, a large workload of grasping tasks is divided into numerous small tasks for each edge device to complete, similar to a multithreaded processing module to process multitudes of files. Usually, network data is acquired by collecting and sorting corresponding web pages. However, this network application layer structure of Hypertext Transfer Protocol (HTTP) mode requires users to send related requests to the Internet end through their network modules. Hence, to access the network data, different from physical data collection, edge devices connected to the Internet are taken as acquisition modules. The web pages containing the required data are found according to a specific algorithm combined with web crawler technology. Then, the overall code of these web pages is downloaded by using the web code download module in the Python environment to complete data collection.

### 4.3. Implementation of Management Algorithm and Construction of Development Environment

With the continuous progress of science and technology, most people have a higher demand for real-time responses to portable devices. However, traditional cloud computing uploads data to the cloud data center for identification and analysis storage, which produces a considerable delay failing to meet the real-time response to data analysis. More importantly, uploading substantial data analysis tasks to the core network simultaneously will bring tremendous pressure to the bandwidth of the core network and even cause network congestion. Therefore, the edge computing technology and the corresponding analysis algorithm are used in parallel to realize the performance appraisal management of the innovation capability of the research team in universities. According to the recognition results and response time, the advantages of the mobile edge computing framework are evaluated for the performance appraisal management of the innovation capability of research teams in universities. The wireless communication rate between the user *UE* and the edge server *S* in the system is calculated as follows:

(7) $$\begin{array}{c} ϒ\left(UE,S\right)=W{\text{.log}}_{2}\left(1+\frac{P^{T}\left(UE,S\right),G\left(UE,S\right)}{\delta^{2}\left(UE,S\right)}\right). \end{array}$$

In equation (7), (*UE*, *S*) represents the communication rate, *P*^*T*^ denotes channel gain, *G* signifies thermal noise power, and *δ*_2_ denotes channel bandwidth. The communication delay between the user equipment *UE* and the server *S* can be estimated by the data transmission volume *D* and the communication rate ϒ(*UE*, *S*), as shown in the following equation:

(8) $$\begin{array}{c} t^{trs}\left(UE,S,D\right)=D.{ϒ}^{-1}\left(UE,S\right). \end{array}$$

### 4.4. Experimental Environment and Model Training Design

The experimental environment here is divided into network training and network testing. The network training equipment is a hardware resource platform based on Titan X GPU, using Xeon E5- 2450@2.00 GHz CPU motherboard with 16 GB memory. The software environment is Ubuntu 16.04 system and Caffe deep learning framework. The experimental environment of the network test part is the NVIDIA Jetson TK1 hardware primary platform, with 2 GB on-board memory. The software environment is Ubuntu 16 of Jetson TK1 customized version 04, Caffe deep learning framework.

MobileNet is trained by transfer learning and the initialized model is pretrained using the ImageNet dataset. ImageNet is an image dataset organized according to the WordNet hierarchy. The ImageNet dataset is meant to illustrate that each synset provides an average of 1000 images. Each concept image is quality-controlled and human-annotated. ImageNet is an ongoing research effort to provide researchers around the world with an easily accessible database of images. Currently, there are a total of 14,197,122 images in ImageNet divided into 21,841 synsets. Rough classification includes amphibian, animal, appliance, bird, covering, and device. Hence, this dataset is the main data source. The training set is divided into multiple batches by batch training method, and the stochastic gradient descent algorithm is used to optimize the model. The batch size is 32. All pictures in the training set are traversed once as an epoch, with a total of 50 iterations, and the initial learning rate is 0.005. The momentum value is 0.9, and then the learning rate is reduced to 0.1 times for every 20 cycles of iteration. The trained model parameter is 3.3 m. In the model experiment, the pruning rate is set to 70%, 80%, and 90%, and the corresponding model parameters are 0.91, 0.58, and 0.23 M. The model parameters are compressed by 3.6, 5.7, and 14.3 times, the quantization accuracy is reduced from 32 bits to 8 bits, and the compression rate is four times.

## 5. Research on Performance Appraisal and Algorithm Optimization

### 5.1. Results Analysis of Innovation Performance Appraisal

The research team of the excellent talent plan of a university in Shaanxi Province is taken as the research object to study the current situation of innovation performance management. The research process mainly conducts research on the performance management of scientific research teams in colleges and universities through questionnaires. The model is then trained through the dataset for research analysis. The research not only conducts effective research on the performance management of scientific research teams in colleges and universities but also provides an important technical reference for the optimization of their performance management.  Figure 5 shows the comprehensive evaluation results and the academic influence of the first-level indicators.

From Figure 5, among six groups, the academic influence scores of Group 1 are the highest. The total index score and academic influence score of Group 2 are slightly lower than those of Group 1, but the program outcome score is significantly lower. The comparison between Group 3 and Group 4 shows little difference in academic influence between the two groups, but there are significant differences in program outcome. There is a slight gap in intellectual force and comprehensive index between Group 5 and Group 4, but the program outcomes of the two groups are the same. Moreover, through the analysis, the academic influence of the team has a specific impact on the comprehensive index of the team, and the relationship between the two shows a positive correlation. On the contrary, the effect of team program outcome on the broad index of the team is not very obvious. Therefore, the proportion of academic influence in the innovation work of colleges and universities is significant, while the proportion of program outcomes is small.  Figure 6 illustrates the comparison results of the academic influence of different research teams.

According to Figure 6, there is a large score gap between the teams with a high level of scientific and technological personnel training and the teams with a general class of scientific and technical personnel training. This shows that there are differences among research teams, and the development of each team in the university tends to be unbalanced. Based on the analysis of their level, each team can arrange development plans according to its characteristics to improve its scientific research level. Group 1 is taken as an example; although Group 1 ranks first, there are specific problems in cultivating scientific and technological talents, which will reduce the scientific research level of the entire research team. Therefore, Group 1 should strengthen the cultivation and introduction of skills.

According to Figures 5 and 6, the uneven development of scientific research teams in different fields in colleges and universities has resulted in a shallow comprehensive impact on the team. Through Figure 7, the scientific research team has made more efforts in the program outcome, but the benefits brought by the program outcome are not high. It may be that the actual value of the program is too low. From this point of view, the scientific research teams in colleges and universities should consider the comprehensive aspects of the research program, focus on the quantity of the research results of the program, and evaluate the quality of the research results. Meanwhile, the ability of academic influence should be strengthened. Compared with the program outcome, literary power accounts for a smaller proportion, which dramatically impacts the improvement of the comprehensive ability of university scientific research teams. It is essential to pay attention to the extensive development of various aspects to improve the full capacity of scientific research teams.

## 6. Algorithm Optimization Research

In the performance management of scientific research teams in colleges and universities, a correct and effective management system can not only save scientific research costs for the team but also maximize the interests of scientific researchers, thus reflecting the scientific research ability and academic influence of the team. Figure 7 shows the identification results of the model constructed on the management level of innovation ability performance assessment of university scientific research teams.

In Figure 7, when the overall compression rate of the model is 14.4 times, the recognition accuracy of the innovation ability performance assessment of the university scientific research team is 95.99%. When the overall compression rate of the model is 22.8 times, the recognition accuracy of the innovation ability performance assessment of the university scientific research team is 95.55%. When the overall compression rate of the model is 57.22 times, the recognition accuracy of the innovation ability performance evaluation of the university scientific research team is 95.55%. Additionally, the values of Precision, Recall, and weighted average score also indicate that the constructed model has high robustness.

The channel-modified model, the track-modified model, and the quantization model are trained with standard multiclass loss functions with modification rates of 70%, 80%, and 90%, respectively, to further test the performance of the edge-side model. In this way, not only can the calculation accuracy of each model be analyzed, but also its comprehensive calculation capability can be studied. The trained hyperparameters are consistent with the training hyperparameters compared to the models reported here.  Figure 8 shows the comparison results of different algorithms under the same conditions, which can better reflect the advantages of the constructed model through analysis.

In Figure 8, under different modification rates, the model has higher model compression rate and recognition accuracy compared to other model compression methods. In addition, the higher the compression rate, the more obvious the improvement in recognition accuracy. Therefore, the model can better analyze the performance evaluation level of innovation ability of scientific research teams in colleges and universities.

## 7. Experiment on Response Time Prediction

Figure 9 shows the experimental results of comparing the prediction times of the proposed system and the backpropagation neural network (BPNN).

The prediction time of the model reported here is compared with that of the backpropagation neural network (BPNN). Under the same conditions, two models read the same data. According to the results in Figure 9, there is no significant difference in the prediction accuracy of the innovation performance of university scientific research teams between this model and BPNN after 20 times of training. Besides, with increasing the amount of training, the performance of this model becomes much better than that of BPNN. Therefore, the model reported here is suitable for predicting scientific research performance in complex scenarios.

## 8. Conclusions

Colleges and universities are the direct embodiment of national innovation ability and one of the main research objects. The innovation ability of colleges and universities determines the country's innovation ability to a large extent. Therefore, firstly, AHP is used to explore the innovation performance appraisal system of scientific research teams. Weight optimization helps to improve the accuracy and rationality of the innovation performance appraisal system of scientific research teams. However, assuming that the output of scientific research results and the number of scientific research projects are equal to the innovation performance of the scientific research team, the team loses the essence of performance evaluation. Therefore, colleges and universities should implement a performance appraisal index system and establish a corresponding reward and punishment system. Then, computer technology and lightweight deep network are used to construct the innovation ability performance evaluation management system of university scientific research team. Various comprehensive tests have been carried out on the performance appraisal management of scientific research teams in colleges and universities. These results make the performance management evaluation of scientific research teams in colleges and universities more comprehensive and reliable and enhance the value of performance evaluation of scientific research teams. On this basis, the essential characteristics of team innovation ability are analyzed. The influencing factors that can improve the innovation ability of scientific research teams in colleges and universities are summarized. Combined with the main problems existing in the innovation ability of scientific research teams in colleges and universities, this study puts forward strategies for improving the innovation ability of scientific research teams in Chinese universities. The designed MobileNet model has a recognition accuracy rate of 95.55% for the performance evaluation of innovation ability of university scientific research teams, which provides an effective management method for the performance management of efficient scientific research teams. Although relatively complete calculation models and methods have been proposed, there is a lack of research on the actual influencing factors, and there is a lack of research on the actual management strategy. In the future research, different university scientific research teams will be selected as the research objects of the field investigation, and a set of operation management strategies will be proposed to enhance the operability of improving the innovation ability of university scientific research teams.

## Figures and Tables

**Figure 1:** The preliminary appraisal index system (part).

**Figure 2:** Important degrees of some indexes.

**Figure 3:** Edge computing system.

**Figure 4:** Edge computing-oriented performance appraisal management method of the innovation ability of university scientific research teams.

**Figure 5:** Comprehensive evaluation results.

**Figure 6:** Academic influence of the first-level index.

**Figure 7:** Performance evaluation results of the innovation ability of university scientific research teams. (a) First test results. (b) Second test results.

**Figure 8:** Comparison of different algorithms. (a) First group. (b) Second group.

**Figure 9:** Comparison of prediction time and experimental results.

## Data Availability

The data used to support the findings of this study are included within the article.
